The article "Application Effect of Doctor-Nurse-Patient Integration Model Based on Heart Rate Management Strategies in Middle-Aged and Young Outpatients with Hypertension" was retracted in 2023. Reasons: unreliable results or conclusions; concerns about the data; concerns about the peer review; concerns about the citations.

# Application Effect of Doctor-Nurse-Patient Integration Model Based on Heart Rate Management Strategies in Middle-Aged and Young Outpatients with Hypertension

**DOI:** 10.1155/2022/7459518

**Published:** 2022-03-16

**Authors:** Jinfang Zhang, Zehong Han, Min Jia, Juanjuan Guo, Hua Guo, Hui Deng

**Affiliations:** ^1^Outpatient Department, HeJi Hospital, Changzhi Medical College, Changzhi, 046000 Shanxi Province, China; ^2^Cardiology of Department, HeJi Hospital, Changzhi Medical College, Changzhi, 046000 Shanxi Province, China

## Abstract

**Objective:**

In this study, a doctor-nurse-patient integration management scheme based on heart rate (HR) management strategies was constructed to explore its application effect in the health management of young and middle-aged outpatients with hypertension.

**Methods:**

A total of 75 young and middle-aged patients with essential hypertension admitted to the Outpatient Department of Cardiology of Heji Hospital Affiliated to Changzhi Medical College, Shanxi Province, from October 2019 to July 2020 were selected and divided into an observation group (*n* = 37) and a control group (*n* = 38) according to different treatment methods. The control group was treated with routine health education, basis on which, the observation group was additionally intervened by the doctor-nurse-patient integration model established upon HR management strategies. The resting heart rate (RHR) awareness, medication compliance, RHR, systolic/diastolic blood pressure (SBP/DBP), and self-management ability were compared between the two groups before and 3 months after intervention. The diet control rate, hypertension awareness rate, and regular review rate were also compared.

**Results:**

The RHR awareness and medication compliance were significantly higher in the observation group compared with the control group after intervention (*P* < 0.05). There were 29 patients with high compliance in the observation group and 19 in the control group, with a significant difference between the two groups (*P* < 0.05). The mean RHR, as well as the mean SBP and DBP in the observation group, were significantly lower than those in the control group (*P* < 0.05). In terms of health behavior assessment, the observation group outperformed the control group in the score of each dimension of self-actualization, health responsibility, stress management, interpersonal support, exercise, and nutrition (*P* < 0.05). In addition, the self-management ability of diet, exercise, medication, blood pressure (BP) monitoring, and disease awareness was significantly higher in the observation group compared with the control group.

**Conclusions:**

For middle-aged and young outpatients with hypertension, the doctor-nurse-patient integration model based on HR management strategies can improve the RHR awareness of patients and improve their medication compliance and self-management ability, thus better controlling the levels of RHR and BP.

The article "Application Effect of Doctor-Nurse-Patient Integration Model Based on Heart Rate Management Strategies in Middle-Aged and Young Outpatients with Hypertension" was retracted in 2023. Reasons: unreliable results or conclusions; concerns about the data; concerns about the peer review; concerns about the citations.

## 1. Introduction

Hypertension, one of the common health problems in the world, has a predilection for the elderly. However, its prevalence in young and middle-aged people has been increasing year by year [1, 2]. The low awareness rate of the disease, poor treatment, and control, as well as the resulting lifelong and high cardiovascular risk, have made it one of the major global public health problems [3]. Studies have confirmed that elevated resting heart rate (RHR) can lead to increased blood pressure (BP) and target organ damage (TOD), increase the incidence of cardiovascular events (CVEs) and mortality in hypertensive patients, and directly damage the cardiovascular system, including increasing myocardial oxygen consumption, accelerating atherosclerosis, reducing plaque stability, and triggering arrhythmia [4]. Therefore, exploring the HR management strategies of young and middle-aged hypertensive patients is of great significance for suppressing the above cardiovascular events and reducing the morbidity in this patient population.

In recent years, the management of HR in patients with hypertension has been increasingly concerned. Hypertension management guidelines in Europe, Taiwan, and other regions all point out the importance of RHR management for hypertensive patients [5, 6]. Therefore, HR management has become a new direction of comprehensive management of hypertensive patients following the control of BP, blood sugar, and blood lipids. Exploring the clinical benefits of HR management in hypertension has gradually become a research hotspot. The current status of HR control in Chinese hypertensive patients is not optimistic. More than 30% of hypertensive patients have a RHR of over 80 beats/min, and this phenomenon is common among the young and middle-aged [4]. The existing studies on HR management mostly focus on medication management to control RHR [7, 8]. However, there are few reports on the education of HR management for this patient population, let alone the awareness of the damage to the cardiovascular and cerebrovascular systems caused by increased RHR. Accordingly, this study is proposed to manage the health of young and middle-aged outpatients with hypertension through the use of a doctor-nurse-patient integration education model based on HR management strategies, so as to strengthen patients' awareness of HR and HR management, and establish good compliance behavior to control HR and BP, which has far-reaching practical significance for the control of hypertension. The novelty of this study lies in the comprehensive evaluation of middle-aged and young outpatients with hypertension from the aspects of RHR knowledge cognition, medication compliance, RHR, systolic blood pressure (SBP), diastolic blood pressure (DBP), diet control rate, hypertension awareness rate, and regular review rate. The report is as follows.

The article "Application Effect of Doctor-Nurse-Patient Integration Model Based on Heart Rate Management Strategies in Middle-Aged and Young Outpatients with Hypertension" was retracted in 2023. Reasons: unreliable results or conclusions; concerns about the data; concerns about the peer review; concerns about the citations.

## 2. Participants and Methods

### 2.1. Research Participants

A total of 75 outpatients with essential hypertension who visited the Vasculocardiology Department in the Heji Hospital Affiliated to Changzhi Medical College, Shanxi Province, from November 2019 to July 2020 were selected. The participants were divided into a control group (*n* = 38) and an observation group (*n* = 37) according to different treatment methods. Inclusion criteria are as follows: ① Patients were diagnosed as essential hypertension based on the National Clinical Practice Guidelines on the Management of Hypertension in Primary Health Care in China [9], with SBP ≥ 140 mmHg and/or DBP ≥ 90 mmHg measured three times under non-same-day resting condition. Those with secondary hypertension such as hyperthyroidism and aortic stenosis were excluded; ② age: 19-64; ③ RHR ≥ 80 beats/min; ④ proficiency in using mobile WeChat platform; ⑤ ability to complete RHR and BP measurements at home; and ⑥ participation in this study on a voluntary basis. Exclusion criteria are as follows: ① severe heart diseases such as thyroid disease, diabetes, resting arrhythmia, sinus block, and myocardial infarction, or liver, kidney, heart, brain, lung, and other diseases; ② those engaging in other similar research; and ③ cognitive or verbal communication disorders. This study has been approved by the Ethics Committee of Heji Hospital Affiliated to Changzhi Medical College and was conducted in accordance with the guidelines laid down in the *Declaration of Helsinki*. All the enrolled patients were willing to participate in this study and signed the informed consent.

### 2.2. Research Methods

All the researchers were specifically involved in the management implemented in the control group and the observation group. Both groups were treated with standardized treatment regimens with balanced doses over the 3 months of intervention.

(1) *Control Group*. Patients received regular postdiagnosis health guidance and telephone follow-up visits. Specifically, at the end of outpatient treatment, the clinic nurses (who are members of the research team) gave health education to patients. In addition, on Friday of the first week of each month, patients were visited by telephone and given educational guidance, mainly including RHR, BP, diet, exercise, medication precautions, and medical guidance
(2) *Observation Group*. On the basis of routine postdiagnosis health guidance, patients were additionally intervened by HR management strategy-based doctor-nurse-patient integration model for health management. The specific scheme is as follows:
  - *Establishment of a Postdiagnosis Team of the HR Management Strategy-Based Doctor-Nurse-Patient Integration Model*. The WeChat group leader (team leader) was headed by the project leader, and the group members were composed of 1 chief cardiologist and 5 nurses. The project leader was in charge of professional knowledge training, and the chief physician of the Department of Cardiology was responsible for answering medical expertise and receiving patients. Three researchers (nurses-in-charge, with a bachelor's degree and more than 10 years of experience in the cardiology ward) were responsible for pushing WeChat messages. WeChat follow-ups of patients in the observation group were organized; 2 investigators (nurse practitioners with a bachelor's degree and more than 5 years of cardiology outpatient service) collected the data of the two groups of patients, established a WeChat group, and guided team members and postdiagnosis patients to scan the QR code to enter the group. Questionnaires were distributed to patients for investigation before and after intervention. All the members of the research team received knowledge training on RHR, hypertension, and related drugs (clinical pharmacists in our hospital were invited to give lectures)
  - *Database Construction of Postdiagnosis RHR Education Knowledge for Young and Middle-Aged Hypertensive Patients*. ① Patients' baseline data such as name, sex, age, RHR, and years and levels of hypertension were collected. ② The project leader, 1 chief cardiovascular physician, and 5 nurses completed the production of RHR education courses or videos, covering RHR detection methods, RHR acceleration, TOD, RHR increase, CVEs, and medication, as well as diet and exercise guidance. In addition, relevant literature was reviewed to develop RHR management education programs
  - *Information System Establishment for Monitoring and Record Keeping and WeChat Platform Set-Up*. A daily patient log sheet was established to monitor the RHR and record the health behaviors of patients. In terms of RHR monitoring and patients' RHR and BP (measured twice a day in the morning and evening, and the mean was calculated) as well as the main symptoms were recorded every day. The health behavior record form was used to record the health behavior measures taken by the patient on a daily basis, such as eating behavior, smoking, drinking, exercise mode, exercise time, drug taking time, and mental health status. In addition, a “doctor-nurse-patient management home of heart rate” was established
  - *Implementation Process*. ① For evaluation of knowledge and behavior, at the end of outpatient visits and routine health guidance, investigators used unified instructions to evaluate patients' HR-related knowledge and medication compliance with questionnaires on the spot, so as to evaluate their mastery of HR-related knowledge and medication compliance. ② For upload of monitoring records, patients were invited to join the WeChat group of “doctor-nurse-patient management home of heart rate” by scanning the QR code face to face. They were required to note their real names in the nickname of the group and set the status of real-time notification for new messages. At the same time, patients were instructed the correct way to measure RHR and BP and were instructed how to fill in the HR and BP monitoring record form and health behavior form (including medication record, diet, exercise, and psychological status), which were photographed and posted to the WeChat group after completion. For those who were unwilling to send the forms to the WeChat group, members of the research team privately added their WeChat to give guidance. ③ For popularization of HR knowledge, targeted education courses were developed according to the evaluation results of patients' knowledge and behavior in the early stage. The project leader pushed HR-related propaganda knowledge in the WeChat group every week in the form of text, audio, and video. The theme of the first month was the basic medical knowledge related to HR, including the concept of RHR, the significance of RHR measurement, the relationship between hypertension and HR, the relationship between HR increase and cardiovascular and cerebrovascular diseases, treatment, and control objectives. The theme of the second month was HR medication education, focusing on monitoring the usage and dosage of medication, mode of administration, drug interaction, etc., in order to improve patients' medication compliance and prevent random drug withdrawal as well as the change and addition of drugs during medication. In addition, patients were encouraged to change their unhealthy habits so as to minimize the effects of nondrug factors on hypertension and drug efficacy. The theme of the third month was HR self-management, including daily diet, exercise, medication, and HR monitoring and management. ④ For online health management, three full-time nurses and 1 chief cardiologist were in charge of checking the daily online records of each patient, to give timely feedback to the patient according to his/her monitoring indicators and the mastery of knowledge related to RHR, BP, and drugs in the questionnaire. Furthermore, relevant education was carried out on the contents that patients had not mastered, so as to urge them to learn by themselves and improve the quality of education. Meanwhile, intervention measures were customized for patients. The medical staff communicated and interacted with patients and provided them with treatment, education, and medical guidance, including lifestyle improvement; monitoring of RHR, BP, and risk factors; guidance on timely medication as directed by doctors; and improvement of unhealthy lifestyle (e.g., sedentary, high-salt diet, smoking, alcoholism, and heavy consumption of coffee and strong tea, which can promote sympathetic nervous excitement and increase the RHR). Moreover, patients were advised to increase physical exercise and aerobic exercise in a planned and gradual manner, aiming to control body weight and improve physical fitness and exercise endurance. Salt control (salt intake < 6 g/d), nonsmoking, and nonalcoholism were also actively encouraged, and those with fast RHR were advised not to drink coffee or strong tea in large quantities, so as to improve their treatment compliance. ⑤ For follow-up evaluation, three months after the implementation of HR management, patients' follow-up visits were reevaluated. Throughout the whole process of online health management, patients' related inquiries and questions were patiently answered one by one. When educating and answering patients' questions, medical staff used plain language and made targeted responses. While receiving education from medical staff, patients can also learn the health behaviors of other patients in the group. At the same time, they can enhance their self-confidence to change bad habits and encourage themselves to follow scientific and healthy behaviors. The flow chart of the nursing process is shown in Figure 1

The article "Application Effect of Doctor-Nurse-Patient Integration Model Based on Heart Rate Management Strategies in Middle-Aged and Young Outpatients with Hypertension" was retracted in 2023. Reasons: unreliable results or conclusions; concerns about the data; concerns about the peer review; concerns about the citations.

### 2.3. Evaluation Indicators

(1) For questionnaire for RHR-related knowledge test, a self-designed questionnaire was used to investigate patients' awareness of RHR-related knowledge and to collect relevant data. There are 10 questions as follows: Question (Q) 1: methods of RHR measurement; Q 2: causes and inducements of RHR increase; Q 3: association between RHR and hypertension; Q 4: association between RHR and diabetes mellitus; Q 5: association between elevated RHR and coronary heart disease; Q 6: association between elevated RHR and stroke; Q 7: association between RHR increase and heart failure; Q 8: dangers of a high RHR; Q 9: an effective lifestyle that lowers RHR; Q 10: target HR of high RHR treatment. One person was counted for each correct answer and 0 for each wrong answer. The content validity index (CVI) of the questionnaire was 0.92, as assessed by 4 medical experts and 1 nursing expert in the Department of Cardiovascular Medicine. The Cronbach's *α* coefficient of the scale was 0.88 in the preexperiment. (2) We used the following four questions to determine patients' compliance with treatment [10]: “Have you ever forgotten to take the medicine? Do you sometimes not take the medicine? Have you stopped taking the medicine after the symptoms have improved? Have you stopped taking the medicine when your condition gets worse?” Patients got 0 points for “yes” and 1 point for “no.” A score of 4 was considered high compliance, 2-3 was considered medium compliance, and 0-1 was considered low compliance. (3) For RHR and BP levels of patients, according to the suggestions in the interpretation of *Chinese Expert Consensus on Heart Rate Management in Hypertension Patients* [4], Omron HEP-907 upper arm sphygmomanometer was used to measure the BP and RHR of patients. Precautions for measurement were as follows: (1) no strenuous exercise, nor coffee, tobacco, or alcohol before measurement; (2) take a comfortable seat with legs not crossed and rest for at least 5 min; (3) keep quiet indoors at room temperature of 18-22 degrees; (4) stay relaxed and stop talking; and (5) keep the center of the cuff at the same level as the heart, with a finger's distance between the arm and the cuff. Two consecutive measurements were made at an interval of one minute. (6) The sphygmomanometer automatically recorded the peak value of pulse wave during the measurement period, calculated the RHR according to the number of pulse waves in the measuring time, and read the readings on the sphygmomanometer dial. The average value was obtained. (7) The Health-Promoting Lifestyle Profile (HPLP) was used to assess the health behaviors of patients from the domains of self-actualization, health responsibility, stress management, interpersonal support, exercise, and nutrition. A total of 52 items were scored by 1-4 scale (1-4 points), with scores proportional to good health behaviors. (4) For self-management ability of patients, we adopted the Chronic Disease Self-Management Program (CDSMP) and conducted the test after adjustment according to the actual situation. The evaluation content included 5 aspects of diet, exercise, medication, BP monitoring, and disease awareness, with a total of 26 items. We used a three-level scoring system, with an overall score of 10 points for each item. The score was proportional to the patient's self-management ability.

The article "Application Effect of Doctor-Nurse-Patient Integration Model Based on Heart Rate Management Strategies in Middle-Aged and Young Outpatients with Hypertension" was retracted in 2023. Reasons: unreliable results or conclusions; concerns about the data; concerns about the peer review; concerns about the citations.

### 2.4. Data Collection Method

After unified training, patients filled in the questionnaire using unified guiding language and following the principle of seeking truth from facts. Before intervention (at the end of the patient's visit) and 3 months after intervention (at the time of patients' return visit), the questionnaire was distributed, and patients were instructed to fill in the relevant survey scales. After filling in and checking that there were no missing items, the questionnaires were collected on the spot. A total of 75 questionnaires were distributed in this study, which were all recovered with an effective recovery rate of 100%.

### 2.5. Statistical Methods

Double entry and validation were used to ensure accuracy of the collected data. The statistical software used in this study was SPSS 23.0 (IBM Corp. Armonk, NY, USA). Measurement data were represented by mean ± standard deviation (($\bar{x}\pm s$)). Independent sample *t*-test was used for intergroup comparisons, and paired *t*-test was used for intragroup comparisons before and after treatment. Count data were expressed as number of cases and percentages (*n* (%)) and compared by *χ*^2^ test. *P* < 0.05 was taken as the level of significance.

## 3. Results

### 3.1. Baseline Data

The general data such as age, sex, educational level, marital status, and course of disease were not significantly different between the two groups, suggesting comparability (*P* > 0.05) (Table 1).

### 3.2. Questionnaire

The comparison of questionnaire evaluation of RHR-related knowledge test between the two groups before and after intervention is shown in Table 2. After intervention, the awareness rate of 10 questions in the questionnaire in the observation group was higher than that in the control group, and the difference was statistically significant (*P* < 0.05).

### 3.3. Medication Compliance and Compliance Degree

The comparison of medication compliance score and compliance degree between the two groups of middle-aged and young hypertensive patients before and after intervention is shown in Table 3. The average score of medication compliance was3.57 ± 0.90points in the observation group and2.89 ± 1.27points in the control group, with a significant difference between the two groups (*P* < 0.05). There were 29 patients with high compliance in the observation group, which was higher than that of 19 cases in the control group (*P* < 0.05).

### 3.4. HR and BP

The comparison of RHR, SBP, and DBP between the two cohorts of young and middle-aged hypertensive patients before and after intervention is shown in Figure 2. The RHR, SBP, and DBP decreased in both groups after intervention, with more significant reductions in the observation group compared with the control group (*P* < 0.05).

The article "Application Effect of Doctor-Nurse-Patient Integration Model Based on Heart Rate Management Strategies in Middle-Aged and Young Outpatients with Hypertension" was retracted in 2023. Reasons: unreliable results or conclusions; concerns about the data; concerns about the peer review; concerns about the citations.

### 3.5. Healthy Behaviors

As shown in Table 4, the observation group was superior to the control group in terms of the total score of health behaviors as well as the score of each dimension of self-actualization, health responsibility, stress management, interpersonal support, exercise, and nutrition (*P* < 0.05).

### 3.6. Self-Management Ability

Finally, we evaluated the self-management ability of the two groups of hypertensive patients after intervention. As shown in Table 5, the observation group was significantly better than the control group in diet, exercise, medication, BP monitoring, and disease awareness (*P* < 0.05).

## 4. Discussion

Given the rising incidence of hypertension among the young and middle-aged, attention should be paid to the management of HR in this patient population [11]. It is well-established that increased RHR is an independent risk factor for hypertension and metabolic disturbances [12]. Higher RHR is associated with increased all-cause mortality and CVEs [13]. Reportedly, there are 245 million people living with hypertension, and the proportion of young and middle-aged patients with hypertension is as high as 67.5% [14]. In addition, the risk of cardiovascular disease in the young and middle-aged increases significantly with the occurrence of hypertension [15–17]. Young and middle-aged people have become the “reserve army” with the rising prevalence of hypertension and the soaring number of cases. Due to busy work, heavy life pressure, and worry about the adverse effects of antihypertensive drugs, middle-aged and young hypertensive patients are not active in antihypertensive treatment and often reduce or stop drugs against the medical advice with poor treatment compliance, resulting in poor control of hypertension [4]. Therefore, attention should be paid to HR education as well as enhancing the awareness of monitoring and managing HR changes, so as to reduce the incidence of CVEs and death risk in young and middle-aged hypertensive patients and improve treatment compliance, thus improving their quality of life.

More and more researchers have explored the application of health management models in patients with hypertension. As reported by Yang et al. [18], the application of health management model based on the perspective of mobile health to hypertensive patients can significantly improve their chronic disease-related health behaviors such as dietary structure, bad living habits, and mental state. Baer et al. [19] proposed that online weight management program integrated with population health management can effectively control the weight of patients with hypertension. In the study of Zhang et al. [20], integrated chronic care models can significantly reduce BP and hospitalization rate in patients with hypertension. In this study, we found that the doctor-nurse-patient integration model based on HR management strategies improved the awareness of RHR in such patient population. In this study, the WeChat platform was used to establish a doctor-nurse-patient HR education group, allowing patients to upload their RHR monitoring records and health behavior records online. In this way, doctors and nurses can not only keep abreast of patients' RHR, BP, symptoms, medication, diet, exercise, and psychological status but also disseminate information about RHR to patients online to facilitate real-time communication and the formulation of personalized treatment and education programs. In addition, patients fed back their postdiagnosis situation in real time through the education platform, allowing medical staff to timely evaluate patients' daily monitoring indicators and behavior habits and give timely feedback, which is helpful for doctors and nurses to dynamically manage patients. On the basis of tripartite interaction of doctors, nurses, and patients, the doctor-nurse-patient integration education model promotes the mutual communication and interaction among the tripartite parties. On the one hand, it can arouse the enthusiasm of patients, improve their attention, and make patients feel humanistic care. On the other hand, this model can give full play to the authority of doctors and make the education content more comprehensive and easier to be accepted by patients, so as to achieve better educational effects [21]. It is shown that the doctor-nurse-patient integrated health education model is conducive to enhancing the self-efficacy and psychological resilience of patients with non-small-cell lung cancer and improving their quality of life [22]. Based on the doctor-nurse-patient integration model, this study carried out comprehensive health management for young and middle-aged hypertensive patients, centering on the initial assessment of knowledge and behavior, patient uploading monitoring records, popularization of HR knowledge, online health management, and later return visit evaluation. The health management has a long duration and rich content. Besides, due to the convenient storage of data on the WeChat platform, patients can refer to and learn the information repeatedly anytime and anywhere, which is convenient for memorizing and improving their knowledge level. Moreover, it can meet the out-of-hospital needs of young and middle-aged hypertensive outpatients. The results in Table 2 of this study show that the observation group had higher awareness of RHR-related knowledge than the control group.

The article "Application Effect of Doctor-Nurse-Patient Integration Model Based on Heart Rate Management Strategies in Middle-Aged and Young Outpatients with Hypertension" was retracted in 2023. Reasons: unreliable results or conclusions; concerns about the data; concerns about the peer review; concerns about the citations.

The doctor-nurse-patient integration model based on HR management strategies can also improve the medication compliance of young and middle-aged hypertensive patients and effectively reduce the RHR and BP levels. Compliance refers to an individual's adherence to the doctor's advice, including medication, diet, exercise, and lifestyle changes. Medication compliance refers to the consistency between the patient's medication behavior and the doctor's advice [23]. Poor drug compliance can be mainly attributed to two reasons as follows: First, due to little disease awareness, patients stop medication on their own when there are adverse reactions [24]; second, poor medication compliance may be caused by the absence of medication guidance, poor doctor-patient communication, inadequate explanation of medication, and/or patients' distrust of medical staff and resistance [25]. With poor self-care awareness, young and middle-aged hypertensive patients may be less willing to accept antihypertensive drug therapy due to high work pressure and the fear of drug side effects, resulting in poor treatment compliance. In this study, the full-time responsible personnel of the research team conducted all-round health knowledge education (hazards of high RHR, mechanism of high RHR hypertension, entry point of high RHR management, treatment of high RHR hypertension, medication knowledge, indications for drug withdrawal, etc.) for patients in the WeChat group every week, which really achieved a breakthrough in time and region, shortened the relationship between doctors and patients, expanded the depth and breadth of health education, and enabled young and middle-aged hypertensive patients to have a deeper understanding of the importance of managing RHR. At the same time, the regular reminder function of the WeChat platform was used to remind patients to take medicine regularly, which urged and supervised the daily health behaviors of patients to take medicine on time and in quantity, helped them establish healthy behavior norms, and improved their medication compliance. The results of this study (Table 3) revealed that after receiving the doctor-nurse-patient integrated education on the basis of HR management, the medication compliance score of patients increased more significantly in the observation group compared with the control group. Moreover, the number of cases with high compliance in the observation group increased significantly, and the number of cases with medium and low compliance decreased. This is similar to the research results of Ai and Zhao et al. [26, 27], demonstrating that the doctor-nurse-patient integration model based on HR management strategies can effectively improve patients' medication compliance. The reasons behind these results may be the following: (1) The patients' HR awareness has been improved through the education of HR-related knowledge. (2) Under this intervention model, the patients' awareness of HR monitoring and management was increased, the healthy codes of behavior were established, and the medication compliance was improved, resulting in effective reductions in RHR and BP levels. As can be seen from Table 4, the health behavior scores of the observation group were significantly higher than those of the control group after intervention. Finally, it can be seen from Table 5 that the self-management ability of patients in the observation group was also significantly stronger than that in the control group, demonstrating the effectiveness and reliability of the application of HR management strategy-based doctor-nurse-patient integration model for patients with RHR.

The article "Application Effect of Doctor-Nurse-Patient Integration Model Based on Heart Rate Management Strategies in Middle-Aged and Young Outpatients with Hypertension" was retracted in 2023. Reasons: unreliable results or conclusions; concerns about the data; concerns about the peer review; concerns about the citations.

However, this study also has some limitations. First, this is a single-center study, with fewer selected research cases and shorter intervention time. Second, the observation outcomes are mainly the awareness of RHR-related knowledge, medication compliance, and the control levels of RHR and BP. However, the health management of young and middle-aged patients with hypertension is a long-term task. Therefore, multicenter research should be carried out in the future to further expand the sample size, prolong the intervention time, and increase the outcome measures. In addition, long-term follow-up data are needed to further confirm the effect of this model in reducing the risk of CVEs.

## 5. Conclusion

To sum up, the results of this study showed that by adopting the doctor-nurse-patient integration model based on RHR management strategies to manage the health of young and middle-aged hypertensive outpatients, patients' awareness of RHR-related knowledge and medication compliance were significantly enhanced, and the RHR, SBP, and DBP levels as well as the self-management ability were significantly improved. Our study not only puts forward new management strategies for middle-aged and young outpatients with hypertension but also provides new insights into the control of patients' conditions and signs.

## Figures and Tables

**Figure 1:** Nursing flow chart.

**Figure 2:** Comparison of heart rate and blood pressure between two groups. The resting heart rate, systolic blood pressure, and diastolic blood pressure of patients in the observation group (*n* = 37) were lower than those in the control group (*n* = 38) (*P* < 0.05). Note: ^∗^*P* < 0.05 between two groups. Independent sample *t*-test was used for intergroup comparison, and paired *t*-test was used for intragroup comparison before and after treatment.

The article "Application Effect of Doctor-Nurse-Patient Integration Model Based on Heart Rate Management Strategies in Middle-Aged and Young Outpatients with Hypertension" was retracted in 2023. Reasons: unreliable results or conclusions; concerns about the data; concerns about the peer review; concerns about the citations.

**Table 1:** Comparison of general data between the two groups ($\bar{x}\pm s$, *n* (%)).

Variables	*n*	Observation group (*n* = 37)	Control group (*n* = 38)	*χ* ^2^/*t*	*P*
Gender				0.024	0.878
Male	48	24 (64.86)	24 (63.16)		
Female	27	13 (35.14)	14 (36.84)		
Age (years)	75	44.44 ± 8.32	46.10 ± 7.75	0.894	0.374
Education level				0.128	0.938
Junior high school and above	13	7 (18.92)	6 (15.79)		
High school/technical secondary school	33	16 (43.24)	17 (44.74)		
Graduate and above	29	14 (37.84)	15 (39.47)		
Occupation				0.205	0.651
Employed	55	28 (75.68)	27 (71.05)		
Nonemployed	20	9 (24.32)	11 (28.95)		
Marital status				0.126	0.722
Married	66	32 (86.49)	34 (89.47)		
Single	9	5 (13.51)	4 (10.53)		
Course of disease (years)				0.162	0.922
2	9	5 (13.51)	4 (10.53)		
2-9	25	12 (32.43)	13 (34.21)		
10	41	20 (54.06)	21 (55.26)		

**Table 2:** Comparison of RHR awareness rate between the two groups before and after intervention (%).

Item	Number of cases with RHR awareness before intervention (*n*/%)		Number of cases with RHR awareness after intervention (*n*/%)	
	Observation group (*n* = 37)	Control group (*n* = 38)	Observation group (*n* = 37)	Control group (*n* = 38)
Question 1	20 (54.1)	22 (57.9)	37 (100.0)^∗∗^	30 (78.9)
Question 2	22 (59.5)	23 (60.5)	37 (100.0)^∗∗^	29 (76.3)
Question 3	16 (43.2)	15 (39.5)	35 (94.6)^∗^	28 (73.7)
Question 4	19 (51.4)	18 (47.4)	33 (89.2)^∗∗^	23 (60.5)
Question 5	19 (51.4)	17 (44.7)	34 (91.9)^∗^	28 (73.7)
Question 6	17 (45.9)	18 (47.4)	32 (86.5)^∗^	25 (65.8)
Question 7	13 (35.1)	14 (36.8)	32 (86.5)^∗^	23 (60.5)
Question 8	21 (56.8)	22 (57.9)	34 (91.9)^∗∗^	24 (63.2)
Question 9	21 (56.8)	22 (57.9)	36 (97.3)^∗∗^	28 (73.7)
Question 10	15 (40.5)	14 (36.8)	37 (100.0)^∗∗∗^	25 (65.8)

RHR: resting heart rate. ^∗^*P* < 0.05, ^∗∗^*P* < 0.01, ^∗∗∗^*P* < 0.001 vs. the control group.

**Table 3:** Comparison of compliance score and compliance degree between the two groups of young and middle-aged hypertension patients before and after intervention ($\bar{x}\pm s$, *n* (%)).

Groups	*n*	Score (point)	High compliance, *n* (%)	Medium compliance, *n* (%)	Low compliance, *n* (%)
Observation group	37	3.57 ± 0.90	29 (78.4)	6 (16.2)	2 (5.4)
Control group	38	2.89 ± 1.27	19 (50.0)	10 (26.3)	9 (23.7)
*t*/*χ*^2^ value		2.669	6.553	1.139	5.005
*P* value		0.009	0.010	0.268	0.025

**Table 4:** Health behaviors of two groups after intervention ($\bar{x}\pm s$).

Categories	Observation group (*n* = 37)	Control group (*n* = 38)	*χ* ^2^ value	*P* value
Total score	121.04 ± 11.75	78.94 ± 7.84	18.298	<0.001
Self-actualization	24.61 ± 3.77	14.01 ± 1.84	21.902	<0.001
Health responsibility	22.03 ± 2.62	16.91 ± 3.36	15.538	<0.001
Stress management	24.77 ± 16.89	13.56 ± 1.92	7.346	<0.001
Interpersonal support	19.84 ± 3.42	15.68 ± 3.45	5.243	<0.001
Exercise	20.86 ± 3.46	15.29 ± 2.20	8.342	<0.001
Nutrition	16.92 ± 2.10	13.36 ± 2.53	6.621	<0.001

The article "Application Effect of Doctor-Nurse-Patient Integration Model Based on Heart Rate Management Strategies in Middle-Aged and Young Outpatients with Hypertension" was retracted in 2023. Reasons: unreliable results or conclusions; concerns about the data; concerns about the peer review; concerns about the citations.

**Table 5:** Self-management ability of patients in the two groups after intervention ($\bar{x}\pm s$).

Categories	Observation group (*n* = 37)	Control group (*n* = 38)	*χ* ^2^ value	*P* value
Diet	8.21 ± 1.30	3.29 ± 1.34	16.133	<0.001
Exercise	7.12 ± 1.08	3.10 ± 0.97	16.969	<0.001
Medication	9.27 ± 0.54	3.97 ± 0.92	30.321	<0.001
Blood pressure monitoring	8.36 ± 1.13	3.29 ± 0.86	21.902	<0.001
Disease awareness	8.43 ± 0.86	2.89 ± 1.02	25.397	<0.001

## Data Availability

The simulation experiment data used to support the findings of this study are available from the corresponding author upon request.
